# Differential Evolution Algorithm with Diversified Vicinity Operator for Optimal Routing and Clustering of Energy Efficient Wireless Sensor Networks

**DOI:** 10.1155/2015/729634

**Published:** 2015-10-01

**Authors:** Subramaniam Sumithra, T. Aruldoss Albert Victoire

**Affiliations:** Anna University, Regional Centre, Coimbatore, Tamilnadu 641047, India

## Abstract

Due to large dimension of clusters and increasing size of sensor nodes, finding the optimal route and cluster for large wireless sensor networks (WSN) seems to be highly complex and cumbersome. This paper proposes a new method to determine a reasonably better solution of the clustering and routing problem with the highest concern of efficient energy consumption of the sensor nodes for extending network life time. The proposed method is based on the Differential Evolution (DE) algorithm with an improvised search operator called Diversified Vicinity Procedure (DVP), which models a trade-off between energy consumption of the cluster heads and delay in forwarding the data packets. The obtained route using the proposed method from all the gateways to the base station is comparatively lesser in overall distance with less number of data forwards. Extensive numerical experiments demonstrate the superiority of the proposed method in managing energy consumption of the WSN and the results are compared with the other algorithms reported in the literature.

## 1. Introduction

In wireless sensor networks, all nodes cooperate to maintain connectivity. These networks are power constrained as nodes operating with limited battery power [1]. Recently it is criticized that the current WSN wastes energy due to an unoptimized network design, which does not consider the energy consumption of network elements such as routers and switches [2]. In general, the design of a routing protocol with multiconstrained metrics has not always taken into consideration the consumption of battery energy. Thus, upon operation of the whole network, some mobile nodes can have problems with energy overhead due to a lack of balance in their battery energy consumption [3, 4].

With the advent of several soft computing techniques, evolutionary algorithms have been widely popular among researchers [5]. A large body of literature conveys that these algorithms have been studied to solve many optimization problems in various disciplines [6–9]. For examples, genetic algorithm (GA) has been applied to enhance the efficiency of construction automation system. Similarly, particle swarm optimization (PSO) has been applied to solve various optimization problems in electrical power. Clustering and routing are two well-known optimization problems which are well researched for developing many nature-inspired algorithms in the field of wireless sensor networks (WSNs) [4]. In [1], the authors have used PSO for clustering and routing in wireless sensor networks. Though PSO is a very efficient optimizer it suffers from curse of dimensionality [10].

The performance of Differential Evolution (DE) has been proved to be outstanding in comparison to the other algorithms tested [11]. It is simple and robust, converges fast, and finds the optimum in almost every run. In addition, it has few parameters to set, and the same settings can be used for many different problems. Previously, the DE has shown its worth on real-world problems, and in this study it outperformed PSO and EAs on the majority of the numerical benchmark problems as well. Among the tested algorithms, the DE can rightfully be regarded as an excellent first choice, when faced with a new optimization problem to solve [11, 12].

This paper presents an application of the Differential Evolution algorithm with an improvised operator called Diversified Vicinity Procedure which still makes the DE to better search for better solution as the problem of interest in this paper is a large dimension one. The paper is further proceeds as follows.  Section 2 formulates the problem of interest, efficient energy routing protocol for WSN.  Section 3 presents an overview of Differential Evolution algorithm subsequently the Diversified Vicinity Procedure. The proposed algorithms and the experimental results are presented in Section 4 and conclusion is in Section 5.

## 2. Problem Formulation

The clustering problem is formulated with the main objective to maximize the lifetime of the network as well as minimize the energy consumption of the sensor nodes [1]. By the network lifetime, we mean the time from the deployment of the WSN till the death of the first gateway. Therefore, network life can be maximized if we can maximize the minimum lifetime of the gateways. Energy consumption of the sensor nodes can be minimized by minimizing the distance between sensor nodes and their corresponding gateways. Let *b*_*ij*_ be a Boolean variable such that [1]. This formulation is simply adopted from

(1) $$\begin{array}{c} b_{ij}=\left\{\begin{array}{cc} 1 & S_{i}⟶g_{j}\;\forall i,j:1\leq i\leq N,\;\;1\leq j\leq M\\ 0 & \text{otherwise}, \end{array}\right. \end{array}$$

where *S* = *s*_1_, *s*_2_,…, *s*_*N*_ is set of sensor nodes.

Let *L* be the minimum lifetime of the gateways; that is, *L* = min⁡{*L*(*i*)∣∀ *i*, 1 ≤ *i* ≤ *M*} and AvegDist be the average distance between sensor nodes and their corresponding CH; that is,

(2) $$\begin{array}{c} \text{AvegDist}=\frac{1}{N}\overset{N}{\underset{i=1}{\sum }}\;\overset{M}{\underset{j=1}{\sum }}\text{dis}\left(S_{i},g_{j}\right)\times b_{ij}. \end{array}$$

*L* denotes the lifetime of the gateway *g*_*i*_. If *g*_*i*_ has residual energy *E*_residual_(*g*_*j*_) and energy consumption per round *E*_Gateway_(*g*_*j*_) then *L*(*i*) can be calculated as follows:

(3) $$\begin{array}{c} L\left(i\right)=\left[\frac{E_{\text{residual}}\left(g_{j}\right)}{E_{\text{Gateway}}\left(g_{j}\right)}\right]. \end{array}$$

Then the Nonlinear Programming (NLP) of the clustering problem can be formulized as follows:

(4) $$\begin{array}{c} \text{Maximize},\;f\left(x\right)=\frac{L\left(i\right)}{\text{AvegDist}}, \end{array}$$

(5) $$\begin{array}{c} \overset{M}{\underset{j=1}{\sum }}b_{ij}=1,\;1\leq i\leq N, \end{array}$$

(6) $$\begin{array}{c} \overset{M}{\underset{j=1}{\sum }}\text{dis}\left(S_{i},g_{j}\right)\times b_{ij}\leq d_{\max},\;1\leq i\leq N,\;\;S_{i}\in S,\;\;g_{j}\in \xi . \end{array}$$

The constraint (5) states that the sensor node *s*_*i*_, ∀*i*  1 ≤ *i* ≤ *N*, can be assigned to one and only one gateway. The constraint (6) ensures that the sensor nodes are assigned to the gateway within its communication range. The set of gateways is denoted by *ξ* = {*g*_1_, *g*_2_,…, *g*_*M*_}. Thus (4) has to be maximized thereby the energy consumption of the cluster heads minimizes.

## 3. Differential Evolution: An Overview

The Differential Evolution (DE), proposed by Storn and Price [12] may be also seen as a simple real-coded GA. The first written article on DE appeared as a technical report in 1995. Since then, DE has proven itself in competitions like the IEEE's International Contest on Evolutionary Optimization (ICEO) in 1996 and 1997, respectively.

In DE community, the individual trial solutions (which constitute a population) are referred as parameter vectors or genomes. DE operates through the same computational steps as employed by a standard EA. However, unlike traditional EAs, DE employs difference of the parameter vectors to explore the objective function landscape. Like other population-based search techniques, DE generates new points (trial solutions) that are perturbations of existing points, but these deviations are neither reflections like those in the CRS and Nelder-Mead methods, nor samples from a predefined probability density function, like those in Evolutionary Strategies (ES) (1966, 2003). Instead, DE perturbs current generation vectors with the scaled difference of two randomly selected population vectors. To produce a trial vector in its simplest form DE adds the scaled, random vector difference to a third randomly selected population vector. In the selection stage, the trial vector competes against the population vector of the same index. Once the last trial vector has been tested the survivors of all the pair wise competitions become permanent for the next generation in the evolutionary cycle. The flowchart of the DE is given in Figure 1.

### 3.1. Diversified Vicinity Procedure: An Overview

The Diversified Vicinity Procedure (DVP) is a relatively recent metaheuristic which relies on iteratively exploring neighborhoods of growing size to identify better local optima. More precisely, DVP escapes from the current local minimum *x* ^*^ by initiating other local searches from starting points sampled from a neighborhood of *x* ^*^ which increases its size iteratively until a local minimum better than the current one is found. These steps are repeated until a given termination condition is met.

This method is inspired from the method adopted in [10] for solving the economic dispatch problem in electrical power systems. Now we discuss the procedural modeling of DVP.

#### 3.1.1. Rules

A finite set of preselected neighborhood structures is denoted with *N*_*k*_  (*k* = 1,…, *k*_max⁡_) and with *N*_*k*_(*x*) the set of solutions in the *k*th neighborhood of *x*. (Most local search heuristics use one neighborhood structure, i.e., *k*_max⁡_ = 1). The stopping condition may be for example, maximum CPU time allowed, maximum number of iterations, or maximum number of iterations between two improvements. Often successive neighborhood *N*_*k*_ will be nested. Observe that point *x*′ is generated in random steps in order to avoid cycling, which might occur if any deterministic rule was used.

#### 3.1.2. Steps of Basic DVP

*Initialization*. Select the set of neighborhood structures *N*_*k*_  (*k* = 1,…, *k*_max⁡⁡_), that will be used in the search; find an initial solution *x*; choose a stopping condition.

*Repeat* the following until the stopping condition is met:

(i) Set *k* ← 1; (2) Until *k* = *k*_max⁡_, repeat the following steps:
(ii) *Shaking.* Generate a point *x*′ at random from the *k*th neighborhood of *x*  (*x*′ ∈ *N*_*k*_(*x*)).
(iii) *Local search.* Apply some local search method with *x*′ as initial solution; denote with *x*′′ the so obtained local optimum.
(iv) *Move or not.* If this local optimum is better than incumbent, move there (*x* ← *x*′′), and continue the search with *N*_1_(*k* ← 1).
(v) Otherwise, set *k* ← *k* + 1.

As a local optimum within some neighborhood is not necessarily one within another, change of neighborhoods can be performed during the local search phase also. In some cases, as when applying DVP to graph theory, the use of many neighborhoods in the local search is crucial.

DVP has been applied to a wide variety of problems both from combinational and continuous problems were based on a particular problem structure. In continuous location-allocation problem the neighborhoods are defined according to the meaning of problem. In bilinearily constrained problems the neighborhoods are defined in terms of the applicability of the successive linear programming approach, where the problem can be partitioned so that fixing the variables in either in set yields a linear problems, more preciously, the neighborhoods of size *k* are defined as the vertices of the LP polyhedral that are *k* pivots away from the current vertex. However, none of the early applications of DVP to continuous problems in general form.

### 3.2. The DVP Algorithm

See Algorithm 1.

The flowchart of the proposed Diversified Vicinity Procedure for DE algorithm is shown in Figure 2. In the next section this proposed algorithm will be experimented on standard test problems.

## 4. Experimental Results

Experiments were performed with the proposed improvised DE algorithm. The experiments were performed with diverse number of sensor nodes ranging from 200 to 700 and 60 to 90 gateways. Each sensor node was assumed to have initial energy of 2 J and each gateway has 10 J.

We have tested our proposed algorithms extensively and depict the experimental results for both the routing and clustering in a combined way. For the sake of simulation we considered two different network scenarios (WSN#1 and WSN#2). Both of them have the sensing field of 500 × 500 m^2^ areas. For the WSN#1, the position of the base station was taken at (500, 250), that is, in a side of the region and for the WSN#2, the position of the base station was taken at (250, 250), that is, in the center of the region. To execute our proposed algorithms, we considered an initial population of 60 particles and the values of PSO parameters are taken same as in [1].

These experiments were carried out using the tabulated methods in Table 1, for the purpose of comparison of the proposed algorithm. The experiments are carried out by varying the sensor nodes and gateways. Thereby four different cases are presented to show the superiority of the proposed Improvised DE over other existing algorithms.

By looking all the Figures from 3 [Fig fig4] [Fig fig5] to6, the proposed algorithm performs better than other algorithms confirming the fact that our derived fitness function takes care about the energy consumption of the normal sensor nodes by reducing the distances between sensor nodes and the gateways.

The performance of the proposed algorithm is shown in Figure 7, is comparable with that of PSO based one in [1]. This implies that our proposed ImpDE have negligible communication and processing overhead; as a result, the performance of security enhanced protocol is comparable with original algorithms. Therefore, we conclude that our proposed DE based system is more efficient in energy and control overhead as compared to the existing systems.

## 5. Conclusion

It is always evident from practical point of view that an energy efficient communication strategy can significantly prolong the lifetime of any wireless sensor networks. Traditionally the clustering and routing problem will be modeled as integer linear program formulation which is computationally intractable for optimal, energy-aware routing in real time WSN. Similarly traditional routing schemes mostly do not consider energy dissipation of the nodes. Hence this research focused on modeling a Nonlinear Programming formulation of these problems with major focus on delivery of total data packets to the base station and energy consumption of the cluster heads. These formulations have been solved using the newly proposed Differential Evolution (DE) algorithm with an improvised search operator. The proposed algorithm has been experimented on several scenarios of WSNs by varying the number of sensor nodes and gateways. The extensive results show that the proposed algorithms perform better than the existing algorithms reported in the literature.

## Figures and Tables

**Figure 1:** Flowchart for the Differential Evolution (DE) algorithm.

**Figure 2:** Flowchart of the proposed Diversified Vicinity Procedure for DE algorithm.

**Figure 3:** Objective function and its convergence characteristics for energy (J) consumption for 200 sensor nodes and 10 gateways.

**Figure 4 fig4:** Objective function and its convergence characteristics for energy (J) consumption for 300 sensor nodes and 40 gateways.

**Figure 5 fig5:** Objective function and its convergence characteristics for energy (J) consumption for 600 sensor nodes and 40 gateways.

**Figure 6:** Objective function and its convergence characteristics for energy (J) consumption for 600 sensor nodes and 60 gateways.

**Figure 7:** Network performance using the various methods.

**Algorithm 1:** 

**Table 1:** Various methods for experiment and their Parameter settings.

Method	Remarks	Parameter settings
GA	Simple [3]	Pop = 100, CR = 0.8, MR = 0.01
PSO	Simple [1]	Pop = 100, *W*_in_ = 0.4, *W*_out_ = 0.9
DE – 1	Rand/1	Pop = 100, CR = 0.8,
DE – 2	Best/1	Pop = 100, CR = 0.8,
DE – 3	Current-to-rand/1	Pop = 100, CR = 0.8,
DE – 4	Current-to-best/1	Pop = 100, CR = 0.8,
ImpDE	Proposed method	Pop = 100, CR = 0.8,
